# N^6^-methyladenosine modification of circMARK2 enhances cytoplasmic export and stabilizes LIN28B, contributing to the progression of Wilms tumor

This article has been retracted.

**DOI:** 10.1186/s13046-024-03113-9

**Published:** 2024-07-11

**Authors:** Guannan Shu, Zhang Zhao, Tianxin Zhao, Changmi Deng, Jiangquan Zhu, Yufeng Han, Minyu Chen, Jiajia Jing, Gaochen Bai, Dian Li, Feng Li, Jing He, Wen Fu, Guochang Liu

**Affiliations:** 1 Department of Urology, Guangzhou Women and Children’s Medical Center, Guangzhou Medical University, Guangzhou Institute of Pediatrics, Guangdong Provincial Clinical Research Center for Child Health, Guangzhou, 510623 Guangdong China; 2 Department of Pediatric Surgery, Guangzhou Women and Children’s Medical Center, Guangzhou Medical University, Guangzhou Institute of Pediatrics, Guangdong Provincial Key Laboratory of Research in Structural Birth Defect Disease, Guangdong Provincial Clinical Research Center for Child Health, Guangzhou, 510623 Guangdong China; 3 Department of Urology, The First Affiliated Hospital of Sun Yat-Sen University, Guangzhou, 510080 Guangdong China; 4 The First Affiliated Hospital, Sun Yat-Sen University, Guangzhou, 510080 China; 5 State Key Laboratory of Virology, Center for Biosafety Mega-Science, Wuhan Institute of Virology, Chinese Academy of Sciences, Wuhan, 430071 China

**Keywords:** Wilms tumor, LIN28B-LET7 pathway, RNA modification, Patient-derived xenograft model

## Abstract

**Background:**

The potential involvement of circular RNAs (circRNAs) and N^6^-methyladenosine (m^6^A) modification in the progression of Wilms tumor (WT) has not been fully elucidated. This study investigates the regulatory mechanisms and clinical significance of m^6^A-modified circMARK2 and its role in WT progression.

**Methods:**

We identified dysregulated circRNAs through deep sequencing and validated their expression by qRT-PCR in WT tissues. The biological functions of circMARK2 were assessed using clone formation, transwell migration, and orthotopic animal models. To dissect the underlying mechanisms, we employed RNA immunoprecipitation, RNA pull-down, dual-luciferase reporter assays, Western blotting, and immunofluorescence and immunohistochemical staining.

**Results:**

CircMARK2, upregulated in WT tissues, was found to be m^6^A-modified and promoted cytoplasmic export. It facilitated WT progression by stabilizing *LIN28B* mRNA through the circMARK2/IGF2BP2 interaction. *In vitro* and *in vivo* studies demonstrated that circMARK2 enhances the malignant behavior of WT cells. Clinically, higher circMARK2 levels in tumor tissues of WT patients were linked to increased tumor aggressiveness and reduced survival rates.

**Conclusions:**

Our study provides the first comprehensive evidence that m^6^A-modified circMARK2 contributes to WT progression by enhancing *LIN28B* mRNA stability, promoting cellular aggressiveness. CircMARK2 emerges as a potential biomarker for prognosis and a promising target for therapeutic intervention in WT, underscoring the clinical relevance of m^6^A modification in pediatric renal cancer.

**Supplementary Information:**

The online version contains supplementary material available at 10.1186/s13046-024-03113-9.

## Backgrounds

Wilms tumor (WT) or nephroblastoma, accounting for approximately 5% of all childhood cancers, is most commonly diagnosed in children and adolescents, contributing to 80% of pediatric renal cancer cases. Its incidence, estimated at 1 in 10,000 children, peaks at around 3 years of age. Annually, around 1500 new WT cases emerge in Europe and North America, with comparatively lower incidences observed in Asia [1]. Advances in medical interventions have enabled disease-free survival rates to exceed 90% [2]. However, a distinct subset of patients presents with less favorable outcomes, particularly those characterized by high-risk histological or biological markers, refractory metastatic disease, or relapsed tumors. The overall survival rate post-relapse stands at approximately 50% [3, 4]. Consequently, a detailed understanding of the biological properties and mechanisms underlying the progression of WT is of critical importance and remains a primary focus in ongoing research.

Circular RNAs (circRNAs), a unique class of endogenous RNA molecules, are formed through back-splicing of precursor mRNA (pre-mRNA) [5]. Their covalently closed-loop structure confers resistance to exonuclease degradation, enhancing their stability compared to linear RNAs. To date, the human genome is known to encode over 100,000 distinct circRNA species [6]. Emerging research underscores the involvement of circRNAs in a variety of human diseases, particularly in the pathogenesis of malignant neoplasms [7]. Functionally, circRNAs are hypothesized to act as microRNA sponges, interact with RNA-binding proteins to form RNA–protein complexes, and even participate in translational processes [8]. In the context of nephroblastoma, most circRNAs identified to date have been implicated in disease initiation and progression, primarily through circRNA-microRNA-mRNA interaction networks [9, 10]. Despite these advances, the potential role of circRNAs as scaffolds in RNA–protein interactions within nephroblastoma warrants further exploration.

N^6^-methyladenosine (m^6^A) represents the first identified and most prevalent modification in mammalian messenger RNAs (mRNAs) and noncoding RNAs (ncRNAs), encompassing circRNAs [11–13]. As a dynamic and reversible RNA modification, m^6^A is pivotal in regulating various biological processes, including RNA degradation and splicing [14]. Emerging evidence suggests that alterations in m^6^A modification play a critical role in tumorigenesis and influence the prognosis of diverse cancers, including those of the colon, lung, pancreas, and prostate [15–17]. Our prior investigations into the molecular epidemiology of WT have identified correlations between genetic polymorphisms in key m^6^A-regulating enzymes, such as METTL14, ALKBH5, YTHDC1, and FTO, and the susceptibility to WT [18–21]. However, the specific impact of m^6^A modification on the aberrations of critical circRNAs, and their consequential roles and mechanisms in the malignant progression of WT, remain underexplored and constitute a significant gap in our understanding.

In this study, we elucidate the pivotal role of a specific circular RNA, circMARK2, in the progression of WT. Our findings reveal that circMARK2, undergoing m^6^A modification, is significantly upregulated in WT and is closely associated with advanced disease stages and poorer survival rates. Utilizing patient-derived xenograft (PDX) models, we demonstrate that enhanced expression of circMARK2 markedly accelerates WT progression. We have uncovered that circMARK2 is exported from the nucleus to the cytoplasm in an m^6^A-dependent manner, mediated by the HNRNPC protein. Crucially, we found that increased cytoplasmic circMARK2 significantly stabilizes *LIN28B* mRNA by interacting with the RNA-binding protein IGF2BP2. This interaction leads to a marked increase in the aggressive behavior of WT cells. Clinically, elevated levels of circMARK2 and *LIN28B* mRNA are more commonly observed in advanced WT tissues, underscoring their potential as prognostic indicators for WT progression. Our results highlight the critical role of circMARK2 in WT pathogenesis and suggest its potential as a therapeutic target for this malignancy.

## Methods

### Care and maintenance of animals

All *in vivo* experiments were approved and performed in strict accordance with the guidelines of the Institutional Animal Care and Use Committee of SYSUCC and Guangzhou Women and Children's Medical Center, Guangzhou Medical University. BALB/c nude mice, aged 3–4 weeks, were procured from Vital River Laboratory Animal Technology Co. Ltd. (China). Additionally, 4–5-week-old male NCG mice (NOD/ShiLtJGpt-Prkdc^em26Cd52Il2rg^em26Cd22/Gpt) were acquired from GemPharmatech Co. Ltd. (China) and maintained in a sterile, pathogen-free environment. To establish the patient-derived xenograft (PDX) model, male NCG mice of 4–5 weeks were engrafted subrenally with primary cells obtained from fresh human Wilms tumor tissue specimens. For the orthotopic rescue assays, sub-capsular injections were performed using cells that had been stably transfected with either a negative control, shRNA, or a circMARK2 overexpression plasmid, with a density of 1 × 10^5^ cells in a 5 μL volume per mouse. Each experimental group comprised five mice, which were randomly assigned. Imaging was executed using the Xenogen IVIS Lumina system, and lung tissues were harvested for hematoxylin and eosin (H&E) staining. In experiments designed to assess the impact of C-SLN nanoparticles (NPs) and circMARK2 knockdown, a sub-capsular WT model was established. Three weeks post-implantation, 15 nude mice were randomly divided into three groups to receive treatments via tail vein injection: naked siRNA, C-SLN NPs, or C-SLN NPs coupled with siRNA. Each mouse received a total dose of 4 μg of siRNA, administered twice weekly over a three-week period. The sample size was determined based on prior empirical knowledge and relevant literature for the specific experiments conducted. No formal sample size calculation was employed. Animals were allocated to different groups using a randomization method; they were first numbered according to body weight, followed by a random number table to assign them to experimental cohorts. Throughout the study, all data was included in the analyses without any exclusion, and the experiment was not blinded.

### WT patient samples

For circRNA expression sequencing, clinical samples were obtained from two pediatric patients exhibiting recurrence and two without recurrence. Each of these patients, aged below two years, presented with Stage I disease and had tumors weighing under 550 g, classified as having a favorable prognosis. Notably, these tumors did not demonstrate loss of heterozygosity at the 1p/16q loci. None of the four patients received preoperative or postoperative radiotherapy or chemotherapy.

For circRNA expression profiling, we obtained 118 paired pathologically diagnosed WT tumor samples from Guangzhou Women and Children's Medical Center and The First Affiliated Hospital of Sun Yat-sen University. Corresponding adjacent noncancerous tissues were acquired approximately ≥ 5 mm away from the tumor site. The clinical features of the WT patients are summarized in Table S1. Regular follow-up was carried out and DFS was determined from the date of surgery to the date of the first evidence of clinical recurrence. Samples used in this study were approved by the Medical Ethics Committee of Guangzhou Women and Children's Medical Center. The informed consent of each patient was obtained.

### Cell lines and cell culture

Human Wilms tumor (WT) cell lines G401 and SK-NEP-1, along with the human embryonic kidney cell line HEK-293 T, were procured from the Cell Bank of the Chinese Academy of Sciences. The WT cell lines, including patient-derived primary cells, were maintained in McCoy's medium (Gibco, China), while HEK-293 T cells were cultured in Dulbecco's Modified Eagle Medium (DMEM) (Gibco, China). Both media were fortified with 10% fetal bovine serum (FBS) (PAN-Seratech, Germany) and 1% penicillin–streptomycin (Biosharp, China). The cell cultures were incubated at 37°C in a humidified atmosphere containing 5% CO_2_. To ensure authenticity and purity, all cell lines underwent short tandem repeat DNA profiling and were routinely screened for mycoplasma contamination, with all tests returning negative results. The cell lines were used for experiments within two months of culture to maintain their physiological relevance.

### Bioinformatics analysis

Data analysis in this study was conducted using R (version 3.4.3), available at https://www.r-project.org/. For the determination of circMARK2's secondary structures, we utilized Mfold (version 2.3). The three-dimensional (3D) structure of circMARK2 was generated using RNA Composer. Molecular docking procedures were performed using the NPDock web server. The 3D crystal structures of protein domains referenced in this study were sourced from the Protein Data Bank. To visualize the docking models and to determine the contact distances between atoms, Discover Studio software was employed.

### RNA interference (RNAi) and transfection

Transient transfection of circMARK2 was carried out using two distinct siRNAs, along with a scrambled siRNA serving as a negative control, all of which were synthesized by RiboBio (China). The siRNAs were introduced into Wilms tumor (WT) cells employing RNAiMAX transfection reagent (Invitrogen, USA), following the manufacturer’s protocol. Functional assays to evaluate the impact of transfection were conducted 48 h post-transfection. Additionally, lentiviral vectors for the knockdown of circMARK2, as well as their corresponding negative controls, were sourced and quality-verified from Genechem (China).

### Plasmid construction

For the circMARK2 over-expression plasmids, circMARK2 cDNA was synthesized and cloned into a pLC5-ciR vector (Geneseed, China). An empty vector served as negative control. Flag-IGF2BP2 WT and truncated plasmids, truncated circMARK2, Flag-HNRNPC WT and mutant plasmids were obtained from Genecreate (China). Plasmids were transfected using Lipofectamine 3000 (Invitrogen, USA), according to the manufacturer’s instructions. *In vivo* bioluminescence imaging was conducted following the injection of cells transfected with vectors containing Gaussia luciferase (Gluc).

### RNA quantitative real-time polymerase chain reaction

Total RNA was extracted utilizing TRIzol reagent (Invitrogen, USA) and quantified using the NanoDrop 2000 spectrophotometer (Thermo Fisher Scientific, USA). For reverse transcription of RNA, PrimeScript RT Master Mix (Takara, China) was employed. Quantitative real-time polymerase chain reaction (qRT-PCR) was performed using SYBR Green SuperMix (Roche, Basel, Switzerland) on a LightCycler 480 system (Roche, Basel, Switzerland). The expression levels of circRNAs and mRNAs were analyzed using the 2^−ΔΔCt^ method. β-actin and U3 were applied as controls in the cytoplasm and nucleus, respectively.

### Western blot

Cellular lysates were prepared using a lysis buffer supplemented with proteinase inhibitor (Beyotime, China) for cells cultured in dishes. The lysates were subjected to incubation on ice for 15 min, followed by centrifugation at 12,000 g at 4°C for another 15 min. Post-centrifugation, supernatants were collected, and protein concentrations were quantified using the BCA Protein Assay Kit (Thermo Fisher Scientific, USA). For electrophoresis, equal amounts of protein samples were loaded onto 10% SDS-PAGE gels, followed by protein transfer onto PVDF membranes. These membranes were blocked with nonfat milk for 1 h at room temperature and then incubated overnight at 4°C with primary antibodies. This was followed by a 1-h room temperature incubation with secondary antibodies. Detection of hybridizations was conducted using high-signal ECL Western Blotting Substrate (Tanon, China) and visualized on a ChemiDoc Touch Imaging System (BIO-RAD, USA). The primary antibodies used for Western blotting included IGF2BP2 (1:1000 dilution, 11601–1-AP, Proteintech, China), LIN28B (1:2000 dilution, ab191881, Abcam, USA), HNRNPC (1:1000 dilution, sc-32308, Santa Cruz Biotechnology, USA), GAPDH (1:1000 dilution, 5174, Cell Signaling, USA), anti-Flag (1:1000 dilution, 8146, Cell Signaling), METTL3 (1:1000 dilution, ab195352, Abcam), and ALKBH5 (1:1000 dilution, ab195377, Abcam). HRP-conjugated secondary antibodies included goat anti-mouse (1:5000 dilution, Proteintech) and goat anti-rabbit antibody (1:5000 dilution, Proteintech).

### Actinomycin D and RNase R treatment

Upon reaching 60% confluence in six-well plates, cells were treated with actinomycin D at a concentration of 5 μg/mL, or with DMSO as a control, and were then harvested at designated time points. Total RNA was subsequently subjected to treatment with 3 U/μg of RNase R (Epicentre Technologies, USA) for 15 min at 37 °C to degrade linear RNAs. Following this treatment, the expression levels of circMARK2 and various mRNAs were quantified using quantitative real-time polymerase chain reaction (qRT-PCR) to assess RNA stability.

### Northern blotting

Custom RNA probes were synthesized by GenePharma (China) for Northern blotting, which was conducted using the NorthernMax Kit (Ambion, Life Technologies, USA) in accordance with the manufacturer’s guidelines. Total RNA, both untreated and treated with RNase R, was separated on a 2% agarose gel and subsequently transferred to a Hybond-N + membrane (GE Healthcare, Sweden) through capillary action. For hybridization, the membrane was incubated overnight at 58°C with biotin-labeled oligonucleotide probes. Detection of these biotin-labeled RNA probes was achieved using the Chemiluminescent Nucleic Acid Detection Module (Thermo Fisher Scientific, USA). GAPDH served as the internal control for these assays, ensuring the accuracy of RNA quantification.

### Nuclear and cytoplasmic extraction

The PARIS Kit (Invitrogen) was used to separate nuclear and cytoplasmic lysates according to the manufacturer’s instructions. Briefly, cells were lysed in Cell Fraction Buffer on ice for 10 min. After centrifugation at 500 × g for 3 min at 4°C, the supernatant was collected as a cytoplasmic fraction. The nuclei were collected followed by washing the pellet with Cell Fraction Buffer.

### Fluorescence in situ hybridization and immunohistochemistry

Oligonucleotide probes specific for circMARK2 and *LIN28B* mRNA were synthesized by GenePharma (China). For fluorescence in situ hybridization (FISH), paraffin-embedded tissue blocks were sectioned into 2.5-μm slices and affixed onto glass slides. FISH was performed on these tissue sections utilizing a FISH kit obtained from GenePharma (China), adhering strictly to the manufacturer's instructions. Imaging of the hybridized sections was carried out using an OLYMPUS FV1000 confocal microscope (Japan), and fluorescence intensity was quantitatively analyzed using ImageJ software. Pearson's correlation coefficient for colocalization studies was calculated using the OLYMPUS FV1000 software. In the immunohistochemistry (IHC) procedures, steps including deparaffinization, rehydration, antigen retrieval, and staining were methodically performed. The normal goat serum blocking buffer (no. ZLI-9056), Rabbit two-step kit (no. PV-6001), and DAB kit (no. ZLI-9017) used in these processes were sourced from ZSGB-BIO (China).

### Immunofluorescence

Cells grown on a confocal dish (Corning, USA) were fixed with 4% paraformaldehyde in PBS for 15 min on ice and then permeabilized with 0.1% TritonX-100 for 10 min. Then, cells were washed twice with PBS and blocked with 5% BSA for 30 min at 37°C. Afterward, cells were incubated with primary antibody overnight at 4°C and washed with PBS. The secondary antibody was incubated for 30 min at 37°C, followed by staining with DAPI for nucleus staining. Fluorescent images were taken with OLYMPUS FV1000 confocal microscopy. Fluorescence densities were analyzed by ImageJ. Correlation analysis was carried out with GraphPad Prism 7 software.

### Transwell assays

Cells were starved for 8 h in serum-free medium. Then, cells were collected, resuspended in serum-free medium, and added to Transwell inserts (Corning, USA). Medium containing 10% FBS was added to the bottom chamber. After incubation for 6–12 h, the migrated cells in lower filters were fixed with 4% polyformaldehyde (Beyotime, China), and stained with 0.4% crystal violet (Beyotime, China) for 20 min. Migrated cells were calculated by capturing five random fields under an Olympus IX83 inverted microscope (Japan). All experiments were performed in triplicate.

### RNA pull-down assays

The biotin-labeled RNA complex was isolated from cell lysates using streptavidin-coated magnetic beads (Invitrogen, Carlsbad, USA). This RNA pull-down procedure was conducted utilizing the Pierce Magnetic RNA–Protein Pull-Down Kit (Thermo Scientific, USA), in strict accordance with the provided manufacturer’s protocol. The presence of target transcripts in the captured fractions was subsequently quantified via quantitative real-time polymerase chain reaction (qRT-PCR). Proteins bound to the biotinylated RNA were then eluted from the beads and subjected to SDS-PAGE analysis. The proteins in the capture complex were identified by western blotting or silver staining or mass spectrometry analysis.

### Silver staining and mass spectrometry analysis

Silver staining was performed with a Fast Silver Stain Kit (Beyotime, China). The targeted region of gel was cut off and saved in microcentrifuge tubes. MS analysis was provided by BGI (Shenzhen, China). A protein presented exclusively in circMARK2 compared to controls, with unique peptides > 2 was considered significant.

### Immunoprecipitation of RNA-binding proteins

RIP was carried out using an EZ-Magna RIP Kit (Millipore, USA) according to the manufacturer's instructions. The m^6^A RIP assay was carried out using a Magna MeRIP m^6^A Kit (Millipore) according to manufacturer's instructions. The rRNAs were removed from the total RNA before the specific enrichment. Five micrograms of IgG, anti-HNRNPC antibody (sc-32308, Santa Cruz Biotechnology) and anti-m^6^A antibody (202003, Synaptic Systems) were used for each sample. The precipitated RNAs were examined through qRT-PCR analyses. The bounded proteins were further confirmed by western blotting.

### Docking simulations, contact maps, and identification of binding site residues

NPDOCK Server was used to determine the possible interaction of circMARK2 with IGF2BP2 and HNRNPC. NPDOCK Server combines GRAMM for global macromolecular docking, scoring with a statistical potential, clustering, followed by refinement of best-scored docked complexes from the three largest clusters. A distance-based approach was used to identify the binding site residues/nucleotides for protein-RNA complexes using a specific cutoff value determined by Discovery Studio.

### Electrophoretic mobility shift assay

Biotin-labeled RNA oligonucleotides were obtained from Umine Biotechnology (Guangzhou, China). The RNA Electrophoretic mobility shift assay (EMSA) was carried out using LightShift™ Chemiluminescent RNA EMSA Kit (Thermo Fisher Scientific, USA), according to the manufacturer’s instructions. Purified proteins were purchased from Origene (USA). For supershift assays, recombinant proteins were pre-incubated with antibodies at 0°C for 20 min followed by the addition of the labeled probe.

### Luciferase reporter assay

The target sequence was cloned separately downstream of the pmirGLO dual luciferase vector (Genecreate, China). Mutations were inserted at the binding sites. Cells were seeded in 24-well plates and transfected with a mixture of pmirGLO dual-luciferase reporter and siRNA at the same time. After 48 h, the relative luciferase activity was measured as the ratio between Firefly and Renilla luciferase activities with a Dual-luciferase Reporter Assay System (Promega, USA). Renilla luciferase activity was used as an internal control. The relative Luc/Rluc ratio was further normalized to that of the control sample in the circMARK2 knockdown or overexpression group.

### Polysome analysis

Approximately 1.5 × 10^7^ cells were incubated in complete medium supplemented with 100 mg/mL cycloheximide (CHX) at 37°C for 10 min prior to cell lysis. Following incubation, the cells were harvested and centrifuged at 1000 × g for 5 min at 4°C. The supernatant was then discarded, and cells were lysed in 500 mL of a specially prepared buffer containing 300 mmol/L NaCl, 20 mmol/L Tris–HCl (pH 7.4), 10 mmol/L MgCl_2_, 1% Triton X-100, 1 mmol/L 1,4-dithiothreitol, 100 mg/mL CHX, 0.5% (w/v) sodium deoxycholate, an EDTA-free protease inhibitor cocktail, and RNase inhibitor. The lysed samples were kept on ice for 10 min. Subsequently, these were centrifuged at 13,000 × g for 5 min at 4°C, and the supernatants were collected for RNA concentration measurements. Sucrose gradient separation was prepared using 5% and 50% sucrose solutions, each containing 100 mg/mL CHX, in a Gradient Master 108 (Biocomp). Equal volumes of cell extracts were layered atop each gradient in ultracentrifuge tubes (Beckman Coulter). The tubes were then centrifuged using a SW41 rotor in a Beckman Coulter Optima™ L-100XP ultracentrifuge at 39,000 rpm for 120 min at 4°C. From these ultracentrifuged tubes, twelve distinct fractions were collected using a Piston Gradient Fractinator (Biocomp). RNA from each fraction was extracted using TRIzol reagent (Invitrogen), and following reverse transcription, quantitative real-time PCR (qRT-PCR) analyses were conducted.

### Statistical analysis

Statistical analyses in our study were conducted using GraphPad Prism 7 software and R software (version 3.4.3), available at https://www.r-project.org/. All experimental procedures were replicated a minimum of three times, with data from a representative experiment presented. Results were expressed as mean ± standard deviation (S.D.). Statistical comparisons among or between groups were carried out using one-way analysis of variance (ANOVA) or independent samples two-tailed Student's t-test. Disease-free survival rates were analyzed via Kaplan–Meier curves, and the Log-rank test was employed to ascertain statistical significance. The correlation between clinicopathological features and circMARK2 expression levels was assessed using the chi-square test. We also calculated the coefficient of variation for these analyses. Hazard ratios (HRs) for univariate and multivariate analyses were determined using Cox regression models. Statistical significance was established at *P* values less than 0.05, with specific levels indicated as follows: *P < 0.05, **P < 0.01, ***P < 0.001.

## Results

### Identification differentially expressed circRNAs in Wilms tumor and characterization of circMARK2

Recent evidence increasingly suggests that circular RNAs (circRNAs) play a pivotal role as signaling regulators in Wilms tumor (WT) [22]. To identify the circRNAs significantly involved in WT, we analyzed a circRNA sequencing dataset (GSE197046), which was derived from WT samples. This analysis revealed 115 circRNAs to be upregulated and 199 circRNAs downregulated in four WT tissues compared to their four paired normal adjacent tissues (NATs), with a threshold of |log2(fold change)|≥ 2 and *p* < 0.05 (Fig. S1A). To further delineate circRNAs integral to WT progression, we conducted circRNA sequencing on primary tumors from two patients with tumor recurrence and two without, as sourced from our institution (Supplementary Data 2). Applying screening criteria for differential expression (|log2(fold change)|≥ 1 and *p* < 0.05) and using circBase for annotation, we shortlisted 77 circRNAs. Intriguingly, of these, 30 circRNAs exhibited upregulation, whereas 47 were downregulated in the tumor tissues of patients at recurrence group in contrast to those at without recurrence group (Fig. 1A). In summary, by intersecting the two aforementioned datasets, we identified four dysregulated circular RNAs as potential candidates for further validation (Fig. 1B, Supplementary Data 2). Among these, hsa_circ_0022614 was notably upregulated in both datasets and exhibited the highest expression level, leading to its selection as our primary research focus. This 234 nt circRNA, hsa_circ_0022614, identified in the human reference genome (GRCh37/hg19), originates from the exon 2 and exon 3 regions of the microtubule affinity regulating kinase 2 (MARK2) gene (chr11:63662630–63663105), and is thus referred to as circMARK2 (Fig. S1B). We observed a significant overexpression of circMARK2 in Wilms tumor cell lines (SK-NEP-1 and G401) compared to the renal epithelial cell line 293 T (Fig. 1C). Divergent primers amplified circMARK2 from complementary DNA (cDNA) but not genomic DNA (gDNA), whereas convergent primers amplified both cDNA and gDNA (Fig. 1D). The unique splice junction of circMARK2 was verified by RT-PCR using divergent primers and Sanger sequencing of the resultant PCR products (Fig. 1E). CircMARK2's resistance to RNase R digestion, as opposed to the sensitivity of *MARK2* mRNA, confirmed its structure as a covalently closed circular RNA (Fig. 1F). Further, qRT-PCR analysis post actinomycin D treatment—a transcription inhibitor—revealed a longer half-life for circMARK2 in WT cells compared to *MARK2* mRNA (Fig. 1G). Subsequently, we used probes that could hybridize with the specific junction to recognize circMARK2, and probes hybridizing with exon 2 to recognize both *MARK2* mRNA and circMARK2, through northern blotting (Fig. 1H). Finally, the cytoplasmic localization of circMARK2 was established through fluorescence in situ hybridization (FISH) (Fig. 1I), corroborating circMARK2's characterization as a typical cytoplasmic circRNA expressed in Wilms tumor.

**Fig. 1:** Differential Expression of circRNAs in Wilms Tumor and Detailed Characterization of circMARK2. **A** Heatmap of high-throughput sequencing between WT with and without recurrence. **B** Volcano plot of circRNAs candidates shortlisted by two datasets. **C** qRT-PCR for the abundance of circMARK2 in different cell lines. Data represent mean ± S.D.; dot plots reflect data points from three independent experiments. **D** Existence of circMARK2 was confirmed by RT-PCR and gel electrophoresis using convergent and divergent primers. CircMARK2 can only be amplified in cDNA. **E** The back-splicing junction was verified by Sanger sequencing. **F** Stability of circMARK2 and linear *MARK2* mRNA assessed by RNase treatment followed by qRT-PCR. Data represent mean ± S.D.; dot plots reflect data points from six independent experiments. **G** Stability of circMARK2 and linear *MARK2* mRNA was assessed by Actinomycin D treatment followed by qRT-PCR at different time points. Data represent mean ± S.D.; dot plots reflect data points from six independent experiments. The *P*-value was determined by two-way ANOVA. **H** Northern blotting of circMARK2 and *MARK2* transcripts by hybridization with exon 2 (left) and junction (right) probes in the presence or absence of RNase R treatment. **I** RNA fluorescence in situ hybridization for circMARK2. Scale bar, 10 µm. **J** Kaplan − Meier analysis of DFS in WT patients with low versus high expression of circMARK2. The *P*-value was determined by a Log-rank test

In our quest to elucidate the relationship between circMARK2 expression and clinical outcomes in WT, we compiled a cohort comprising 118 WT patients (Supplementary Data 3). The expression levels of circMARK2 in 118 paired WT tissues and corresponding adjacent normal tissues were quantified using qRT-PCR. Our analysis revealed a significant upregulation of circMARK2 in WT tissues compared to adjacent normal tissues (Fig. S1C). Moreover, we observed a notable association between circMARK2 expression and higher risk categories as per the revised SIOP or COG working classification [23] (Table S1). Additionally, a significant correlation was established between elevated circMARK2 expression and reduced disease-free survival (DFS) (Fig. 1J). Both univariate and multivariate Cox regression analyses underscored high circMARK2 expression as an independent predictor for recurrence within our WT patient cohort (Table S2). Based on these findings, we hypothesize that circMARK2 may play a crucial role in the pathogenesis and advancement of WT.

### CircMARK2 promotes the proliferation, invasion, and migration of WT cells *in vitro* and *in vivo*

In light of the significant association between circMARK2 expression levels and prognostic indicators in WT, we embarked on a series of *in vitro* and *in vivo* functional assays to elucidate the role of circMARK2 in WT cells. Lentiviral short-hairpin RNAs (sh-circMARK2) were employed to specifically knock down circMARK2 in the G401 cell line, which exhibited higher baseline levels of circMARK2. We used two distinct shRNAs (sh-1 and sh-2) targeting circMARK2 for knockdown. The sh-ctrl represents the control group for the sh-circMARK2 lentiviral vectors. Conversely, we enhanced circMARK2 expression in the SK-NEP-1 cell line, known for its relatively lower circMARK2 expression, by stable transfection with overexpression plasmids (p-circMARK2). Notably, these manipulations did not alter the expression levels of MARK2 mRNA in either cell line (Fig. 2A). Silencing circMARK2 significantly hindered the proliferation of WT cells, observed both *in vitro* and *in vivo* (Fig. 2B, C). Among the two shRNAs, sh-2 exhibited superior knockdown efficiency and a more pronounced effect on cell proliferation compared to sh-1. Therefore, in subsequent experiments, we used only sh-2 for stable knockdown and referred to this as sh-circMARK2 for simplicity. Conversely, overexpression of circMARK2 led to a slight increase in cell proliferation, possibly due to the already high endogenous levels of circMARK2 in these cells (Fig. 2B, C). Transwell assays demonstrated that cell migration was inhibited following circMARK2 knockdown, whereas its overexpression promoted migration (Fig. 2D). Additionally, *in vivo* lung metastasis models, established via tail vein injection of stably transfected cells, revealed a marked decrease in metastatic lung nodules in the sh-circMARK2 group compared to controls. In contrast, an increase in metastasis was observed in the p-circMARK2 group (Fig. 2E). Collectively, these findings underscore the influential role of circMARK2 in modulating the proliferation and invasive capabilities of WT cells.

**Fig. 2:** CircMARK2's Role in Enhancing Proliferation, Invasion, and Migration of Wilms Tumor Cells. **A** RT-PCR analysis of circMARK2 expression and *MARK2* mRNA expression in knockdown (left) or overexpression (right) cell lines. Data represent mean ± S.D.; dot plots reflect data points from three independent experiments. The *P*-values were determined by Student’s t test. **B** Representative images of clone formation assays of indicated WT cells (*n* = 5 per group). Data represent mean ± S.D.; dot plots reflect data points from five independent experiments. The *P*-values were determined by Student’s t test. **C** Representative images of tumors and growth curves of indicated WT cells *in vivo* (*n* = 5 per group). **D** Transwell assays showed that expression of circMARK2 affected the migration ability of WT cells. Top, transwell representative images. Scale bar, 100 µm. Bottom, numbers of migration cells (*n* = 5/group). Data represent mean ± S.D.; dot plots reflect data points from five independent experiments. The *P*-values were determined by Student’s t test. **E** Bioluminescent in the lungs and tumor metastasis formed in the lungs of mice through tail vein injection showed that expression of circMARK2 affected WT metastasis *in vivo*. Left, representative bioluminescent images of lungs for each experimental group. Right, representative lung and representative HE staining of lung metastatic lesions. Scale bar, 100 µm. (*n* = 6 mice/group). The *P*-values were determined by Student’s t test

### CircMARK2 interacts with IGF2BP2 through specific binding sequence

To elucidate circMARK2's functional role in WT, our initial approach involved the use of TransCirc [24], a specialized database assessing the translation potential of circular RNAs. Despite detecting ORF and IRES sequences, proteomic analysis via mass spectrometry and translation initiation site exploration indicated a lack of translation potential for circMARK2. Given recent reports highlighting the significance of circRNA-protein interactions in cancer progression [25, 26], we employed RNA pull-down followed by mass spectrometry (MS) to identify proteins potentially interacting with circMARK2. Notably, HNRNPC and IGF2BP2 were significantly enriched in circMARK2 junction site-targeted probe complexes (Fig. 3A, Table S3). IGF2BP2, an RNA-binding protein, is known to regulate transcript translation by recruiting them to cytoplasmic protein-RNA complexes [27]. Subsequent RNA-binding protein immunoprecipitation (RIP) assays corroborated the enrichment of circMARK2 in IGF2BP2-bound complexes, in contrast to control IgG, in both SK-NEP-1 and G401 cell lines (Fig. 3B). Further RNA pull-down assays, employing cells transfected with shRNAs targeting circMARK2 and a control, showed that circMARK2 knockdown did not affect total IGF2BP2 protein levels, but did diminish the amount of IGF2BP2 bound to circMARK2 (Fig. 3C). Immunofluorescence coupled with fluorescence in situ hybridization (IF-FISH) assays confirmed the cytoplasmic co-localization of circMARK2 and IGF2BP2 (Fig. 3D, Table S4). To delineate which domain of IGF2BP2 was involved in binding circMARK2, we engineered IGF2BP2 mutants with individual KH domain truncations (Fig. S1D). RIP assays in WT cells identified the KH3-4 domain as the specific binding site for circMARK2 (Fig. 3E). To pinpoint the critical circMARK2 sequence for RNA–protein interaction, we performed a computational analysis of circMARK2 interaction with IGF2BP2 (Fig. S1E). To determine the secondary structures of circMARK2, we used the minimum free energy algorithm implemented in Mfold [28]. The secondary structure with a lower theoretical value of free energy was selected as the model structure for the prediction of the three-dimensional (3D) structure (Fig. 3F). The output file containing a primary sequence and an associated secondary structure (Dot-Bracket Notation) was then submitted to RNA Composer to generate the 3D structure [29, 30] (Fig. 3G). The docking procedure between the circMARK2 and IGF2BP2 KH3-4 domain was carried out by the NPDock web server [31]. The 3D crystal structure of IGF2BP2 KH3-4 domain was derived from Protein Data Bank entry 6ROL [32]. The molecular docking output included the best scored structures that were taken from the three largest clusters. The best scored structures showed the interacting sequence of circMARK2 was 5'- AGACUCA-3' (Fig. 3H). All favorable bonds were acquired through Discover Studio. The MC score between circMARK2 and the IGF2BP2 docking domain supported the conclusion that circMARK2 sufficiently docked IGF2BP2 (Fig. S1F). *In vitro* RNA-EMSA confirmed the specific binding of IGF2BP2 to this sequence, with increasing IGF2BP2 concentrations correlating with higher circMARK2/IGF2BP2 complex formation. Mutation of the AGACUCA motif notably reduced this interaction (Fig. 3I). Further evidence that the IGF2BP2 protein binds to the predicted sequence was obtained by employing constructs that overexpressed full-length circMARK2, mutant circMARK2 (circMARK2 MUT) or truncated circMARK2 lacking the former (circMARK2Δ) predicted binding sequence. We transfected the constructs into 293 T cells, and 48 h later performed RNA pull-down assays. In line with earlier results, IGF2BP2 was more enriched in pulldowns from cultures expressing full-length circMARK2 than in cultures expressing circMARK2 MUT or circMARK2Δ (Fig. S1G). Our comprehensive analysis thus demonstrates that circMARK2 interacts with IGF2BP2 through its KH3-4 domain.

**Fig. 3:** Interaction Between circMARK2 and IGF2BP2. **A** Left, identification of the circMARK2-protein complex pulled down by circMARK2 junction probe with protein extracts from WT cells. Right, MS of circMARK2 binding proteins. **B** RIP assays showed the association of IGF2BP2 with circMARK2. Relative enrichment representing RNA levels associated with IGF2BP2 compared to input control. IgG antibody served as a control. Data represent mean ± S.D.; dot plots reflect data points from three independent experiments. **C** Western blotting assay showing the level of IGF2BP2 protein pulled down by biotin-labeled circMARK2 probes from the lysates of WT cells following transfection with shRNAs targeted circMARK2 and negative control. **D** IF-FISH assay showing that circMARK2 is colocalized with IGF2BP2 protein in the cytoplasm. Scale bar, 10 µm. **E** Relative enrichment represented circMARK2 levels associated with truncated IGF2BP2 relative to input control. Data represent mean ± S.D.; dot plots reflect data points from three independent experiments. **F** 2-D RNA structure of circMARK2 generated by Mfold. **G** The 3-D structure of circMARK2 was generated by RNA Composer. **H** Graphical representation of the best three-dimensional structures of circMARK2 and IGF2BP2 (KH3-4 domain) docking models with a zoom-in image. **I** RNA-EMSA assay showing the binding ability of purified IGF2BP2 with wild-type or mutant biotin-labeled oligonucleotides containing predicted sequences from circMARK2

### CircMARK2 guided IGF2BP2 binding and promoting *LIN28B* expression

Given the critical role of IGF2BP2 in mRNA stability and translation [33, 34], we explored whether the circMARK2/IGF2BP2 complex might stabilize downstream targets. RNA sequencing analysis was performed on WT sh-ctrl cells and sh-circMARK2 cells, revealing a significant reduction in 122 mRNAs upon circMARK2 silencing (|log2(fold change)|≥ 2, *p* < 0.05). Considering IGF2BP2's affinity for mRNAs with high AU content [34, 35] we screened these downregulated mRNAs against published RBP CLIP-SEQ datasets, including Starbase [36], and CLIPdb [37], identifying six IGF2BP2-bound mRNAs, including *SLC7A2*, *CKB*, *TSHZ2*, *NCKAP5*, *LIN28B* and *SPRY4*. Given that circMARK2 promotes the progression of WT, *LIN28B*, which encodes a protein that has been mechanistically tied to Wilms tumor development [38], caught our attention. We confirmed that *LIN28B* were abundantly expressed in WT cell lines, and targets of circMARK2 through qPCR and western blotting validation (Fig. 4A, B). Subsequently, through sequence BLAST analysis, we found that the CCAGCAGUAA site of circMARK2 could perfectly bind to the 3′UTR region of *LIN28B* mRNA at the UUACUGCUGG site (Fig. 4C). The interaction was confirmed by separate RNA pull-down assays in WT cell lines (Fig. 4D). Next, we found that the downregulation of circMARK2 significantly suppressed the stability of *LIN28B* mRNA in WT cell line. While overexpression of circMARK2 enhanced the stability of *LIN28B* mRNA (Fig. 4E). Besides, we performed polysome fractionation analyses to determine whether circMARK2/IGF2BP2 influences the translation efficiency of all or specific targeted mRNAs. Our findings indicated that circMARK2 depletion did not impact global polyribosome formation (Fig. 4F). Furthermore, we conducted RT-qPCR on each polysome fraction in control and circMARK2-depleted cells, revealing a leftward shift in the distribution of *LIN28B* mRNA on the fractionation gradient (Fig. 4G). This observation suggests that *LIN28B* mRNA were associated with smaller polysomes upon circMARK2 depletion, implying a suppression of *LIN28B* mRNA translation efficiency due to lower mRNA stability. Consistent with previous studies [32] which reported that KH3-4 was the primary RNA binding domain in IGF2BP2, our RIP assays with IGF2BP2 mutants confirmed that KH3-4 were also responsible for IGF2BP2 and *LIN28B* mRNA binding (Fig. 4H). This finding led us to propose that circMARK2 may act as a mediator between IGF2BP2 and *LIN28B* mRNA.

**Fig. 4:** CircMARK2 Facilitates IGF2BP2 Binding and Upregulates *LIN28B* Expression. **A**, **B** PCR (**A**) as well as Western blotting (**B**) validation of LIN28B upon circMARK2 knockdown and overexpression. **C** Schematic illustration of the binding between *LIN28B* mRNA and circMARK2. **D** Relative enrichment representing *LIN28B* mRNA levels associated with circMARK2 compared to controls. Data represent mean ± S.D.; dot plots reflect data points from six independent experiments. The *P*-values were determined by Student’s t test. **E** Stability alteration of *LIN28B* mRNA upon circMARK2 knockdown or overexpression. **F** Representative traces of polyribosome profiles obtained from sh-Ctrl or sh-circMARK2 cells. **G** RT-qPCR analysis of *LIN28B* mRNA levels in each fraction obtained from sh-Ctrl or sh-circMARK2 cells. **H** Relative enrichment represented the enrichment of *LIN28B* mRNA associated with the truncated IGF2BP2 protein complex compared to the input control. IgG antibody served as a control. Data represent mean ± S.D.; dot plots reflect data points from three independent experiments. **I** IF-FISH assay showed that the colocalization of IGF2BP2/*LIN28B* mRNA was decreased upon knockdown of circMARK2. Scale bar, 10 µm. **J** Relative luciferase activity of luciferase reporter gene with LIN28B-WT or LIN28B-Mut. Data represent mean ± S.D.; dot plots reflect data points from three independent experiments. The *P*-value was determined by Student’s t test. **K** Upon knockdown or overexpression of circMARK2, relative luciferase activity of luciferase reporter gene with LIN28B-WT or LIN28B-Mut. Data represent mean ± S.D.; dot plots reflect data points from three independent experiments. The *P* value was determined by Student’s t test. **L** Upon knockdown or overexpression of circMARK2, relative enrichment representing *LIN28B* mRNA levels associated with IGF2BP2 protein complex compared to the input control. IgG antibody served as a control. Data represent mean ± S.D.; dot plots reflect data points from three independent experiments

Supporting this hypothesis, RNA-FISH assays showed decreased colocalization of IGF2BP2 and *LIN28B* mRNA in circMARK2-knockdown cells, with no change in IGF2BP2 protein levels (Fig. 4I). CircMARK2 overexpression slightly enhanced their colocalization in WT cells (Fig. S2A). Additionally, luciferase reporter assays with wild-type and mutant LIN28B constructs (LIN28B -WT and LIN28B -MUT) revealed that the mutant had significantly lower luciferase activity compared to the wild-type, underscoring the specificity of the interaction (Fig. 4J). Furthermore, circMARK2 knockdown significantly suppressed the expression of luciferase mRNA and luciferase activity of wild-type luciferase reporters, rather than mutant luciferase reporters. In contrast, overexpression of circMARK2 significantly elevated the expression of luciferase mRNA and luciferase activity of wild type luciferase reporters, but not that of mutant luciferase reporters (Fig. 4K). Finally, RIP assays demonstrated that circMARK2 knockdown reduced, and overexpression increased, the enrichment of mRNA in IGF2BP2-immunoprecipitated complexes (Fig. 4L). These findings collectively establish circMARK2 as a key facilitator in the interaction between IGF2BP2 and *LIN28B* mRNA, forming a critical ternary complex.

### CircMARK2 promotes progression of WT through the *LIN28B/LET-7* pathway

*LIN28B*'s association with pluripotency, stem cell renewal, extended kidney development, and Wilms tumor formation via the dysregulation of *LET-7* miRNA biogenesis is well-established [39]. *LET-7*, recognized as a tumor suppressor, targets genes involved in cell cycle regulation, signaling, and maintenance of differentiation [40]. Thus, we conducted Gene Set Enrichment Analysis (GSEA: Human Gene Set: BOYERINAS_ONCOFETAL_TARGETS_OF_LET7) and found *LET-7* target signature genes were down-regulated upon circMARK2 knockdown, including *HMGA2*, *MYC*, and *SLC25A24* (Fig. 5A). Gene Ontology (GO) analysis indicated significant alterations in several *LET-7* associated pathways, such as cell junction and cell differentiation, following circMARK2 silencing (Fig. S2B). We then investigated if the role of circMARK2 in progression of WT is dependent on the *LIN28B*/*LET-7* pathway. In order to more accurately recapitulate the tumor growth characteristics observed in WT patients, we executed a rescue experiment utilizing an orthotopic *in vivo* patient-derived xenograft (PDX) model. This model was established through a sub-capsular injection of primary cells. These cells, sourced from patients with recurrence, were stably transfected with either negative control, shRNA, or a plasmid facilitating the overexpression of the target gene, with an injection density of 1 × 10^5^ cells in a 5 μL volume per mouse. This model revealed that reduced proliferation of WT tumors formed by circMARK2-knockdown cells was substantially reversed by *LIN28B* overexpression (Fig. 5B). Additionally, prolonged observation of tumor-bearing mice showed fewer instances of pulmonary metastasis in the circMARK2 knockdown group compared to controls. Interestingly, circMARK2 knockdown coupled with *LIN28B* overexpression resulted in more metastasis cases in this model (Fig. 5C). *In vitro* assays, including clone formation and transwell assays, corroborated that *LIN28B* overexpression functionally compensated for the decreased cell proliferation and invasion following circMARK2 silencing (Fig. 5D, E). Moreover, the overexpression of a circMARK2 mutant lacking *LIN28B* binding ability led to reduced proliferation and invasion, demonstrating endogenous competition (Fig. S2C, D). *In vitro*, circMARK2 knockdown in WT cells decreased *LIN28B* expression and increased *LET-7* levels, while overexpression of circMARK2 produced the opposite effects (Fig. 5F, G). The elimination of *LIN28B* mRNA in WT cells successfully reversed the effect of circMARK2 overexpression, which led to reduced expression of *LET-7*. *LIN28B* overexpression rescued the effect of circMARK2 knockdown (Fig. 5G). We next compared the *in vivo* expression levels of *LIN28B* and *LET-7* between mice injected with control or circMARK2-silenced PDX cells. We found that downregulations of *LIN28B* and upregulations of *LET-7* were consistent with that of circMARK2 silencing (Fig. S2E). Further analysis of primary tumor and corresponding lung metastasis tissues in the PDX models demonstrated a consistent pattern: an upregulation of *LIN28B*, accompanied by a downregulation of *LET-7* in metastatic tissues (Fig. 5H). These findings imply that within the diverse cellular milieu of the WT PDX model, cell populations characterized by high circMARK2 and *LIN28B* expression, coupled with low *LET-7* expression, are likely the predominant drivers of metastasis.

**Fig. 5:** The Role of circMARK2 in Wilms Tumor Progression via the *LIN28B/LET-7* Pathway. **A** GSEA analysis of *LET-7* pathway upon circMARK2 expression alteration. **B**, **C** PDX models showed that circMARK2 promoted the progression ability of WT cells depending on *LIN28B* expression. **B** Representative images of the orthotopic PDX assay. **C** Tumor metastasis formed in the lungs and bone of the orthotopic PDX assay (*n* = 5/group). **D**, **E** Clone formation assays and transwell assays showed that circMARK2 promoted the progression ability of WT cells depending on *LIN28B* expression. **D** Representative images of the clone formation assays. **E** Representative images of the Transwell assay. Scale bar, 100 µm. (*n* = 3/group). **F** qPCR analysis of *LIN28B* expression upon overexpression or knockdown of circMARK2 in WT. Data represent mean ± S.D.; dot plots reflect data points from three independent experiments. **G** qPCR analysis of *LET-7* expression upon circMARK2 and *LIN28B* simultaneously alteration in WT. Data represent mean ± S.D.; dot plots reflect data points from three independent experiments. **H** qPCR analysis of *LIN28B*, and *LET-7* in primary tumor and metastatic tissues from PDX model. Data represent mean ± S.D.; dot plots reflect data points from three independent experiments. **I** Correlation between circMARK2, *LIN28B* levels and *LET-7* levels in our 118 patient’s cohort. **J** Kaplan − Meier analysis of DFS in WT patients with low versus high expression of *LIN28B*. The *P*-value was determined by a Log-rank test

Exploring the clinical implications of circMARK2 in WT, we evaluated its expression in a cohort of 118 WT patients, finding a positive correlation between circMARK2 and *LIN28B* levels and a negative correlation with *LET-7* levels (Fig. 5I). Notably, the expression levels of *LIN28B* also predicted WT patient DFS (Fig. 5J). Both circMARK2 and *LIN28B* were notably higher expressed in advanced stages of WT and recurrent WT (Table S5). These results collectively suggest that circMARK2's oncogenic role in promoting WT progression is mediated through the *LIN28B*/*LET-7* pathway.

### HNRNPC mediates m^6^A modified circMARK2 cytoplasmic export

HNRNPC, a member of the HNRNP subfamily of RNA binding proteins, plays critical roles in pre-mRNA processing, RNA transport, and m^6^A regulation [41, 42]. Our RNA-binding protein immunoprecipitation (RIP) assays demonstrated significant enrichment of circMARK2 in HNRNPC antibody precipitates compared to control IgG in both SK-NEP-1 and G401 cell lines (Fig. 6A). Subsequent RNA pull-down assays in cells transfected with shRNAs targeting circMARK2 and a negative control revealed that circMARK2 knockdown did not affect total HNRNPC protein levels but reduced its binding to circMARK2 (Fig. 6B). Considering HNRNPC's role as an m^6^A reader, we investigated the presence of m^6^A methylation on circMARK2. Utilizing the sequence-based N^6^-methyladenosine modification site predictor SRAMP [43], we identified the GAACU m^6^A motif as potentially crucial for m^6^A modification (Fig. 6C). Further, we conducted methylated RNA immunoprecipitation (MeRIP) assays, and we precipitated several known m^6^A-containing RNAs (such as *RARA* [44], Fig. 6D). We found that 5’-GAACU-3’ sequence of circMARK2 was also highly enriched in the m^6^A precipitated fraction (Fig. 6D), confirming the m^6^A modification in circMARK2. By browsing the aforementioned computational analysis of circMARK2 interaction with HNRNPC, we identified that GAACU motif is also a putative binding motif between HNRNPC and circMARK2 (Fig. S2F). RNA electrophoretic mobility shift assays (RNA-EMSA) indicated that mutation of the GAACU m^6^A motif in circMARK2 reduced its binding affinity to HNRNPC (Fig. 6E). Furthermore, once mutated the RNA binding motif of HNRNPC, the interaction ability with circMARK2 was decreased (Fig. 6E). These results indicated that HNRNPC interacted with circMARK2 with the m^6^A-binding motif at the GAACU m^6^A motif of circMARK2.

**Fig. 6:** HNRNPC Mediation of m^6^A-Modified circMARK2 for Cytoplasmic Export. **A** RIP assays showed the association of HNRNPC with circMARK2. Relative enrichment representing RNA levels associated with HNRNPC compared to input control. IgG antibody served as a control. Data represent mean ± S.D.; dot plots reflect data points from three independent experiments. **B** Western blotting assay showing the level of HNRNPC protein pulled down by biotin-labeled circMARK2 probes from the lysates of WT cells following transfection with shRNAs targeted circMARK2 and negative control. **C** Schematic illustration showing predicted m^6^A modified site in circMARK2 by SRAMP. **D** MeRIP assay showing that circMARK2 was highly recruited in m^6^A precipitated fraction. Data represent mean ± S.D. from three independent experiments; dot plot reflects data points from independent experiment. The *P*-values were determined by a two-tailed paired Student’s t test. **E** RNA-EMSA assay showing the binding ability of purified HNRNPC with biotin-labeled oligonucleotides containing GAACU motif from circMARK2. **F** Western blotting analysis of WT cells after transfection with vector control, METTL3 or ALKBH. **G** Left panel: MeRIP-qPCR analysis showing enriched circMARK2 after overexpression of METTL3 in WT cells (*n* = 3). Right panel: MeRIP-qPCR analysis showing decreased circMARK2 after overexpression of ALKBH5 in WT cells (*n* = 3). **H**, **I** Cytoplasmic and nuclear RNA fractionation experiment (**H**) and RNA fluorescence in situ hybridization (**I**) showing that knockdown of HNRNPC increased the nuclear circMARK2 content, whereas the dysregulation of nuclear circMARK2 caused by HNRNPC RNAi was recovered by overexpression of WT but not the mutant of HNRNPC. Data represent mean ± S.D. from three independent experiments; The *P*-values were determined by a two-tailed unpaired Student’s t test. **J** MeRIP assay showing that m^6^A methylation levels was increased upon circMARK2 overexpression. Data represent mean ± S. D. from three independent experiments; dot plot reflects data points from independent experiment. The *P*-values were determined by a two-tailed unpaired Student’s t-test. **K**, **L** Clone formation assays (**K**) and Transwell assays (**L**) showing that overexpression of circMARK2 m^6^A-binding mutant attenuated WT cells proliferation and invasion activity. Data represent mean ± S. D. from three independent experiments; dot plot reflects data points from independent experiment. The *P*-values were determined by a two-tailed unpaired Student’s t-test

Given the importance of METTL3 (N^6^-adenosine-methyltransferase) and ALKBH5 (RNA demethylase) in m^6^A modification [45] and their link to Wilms tumor susceptibility [19, 46], we conducted MeRIP following overexpression of these enzymes (Fig. 6F). MeRIP-qPCR after METTL3 and ALKBH5 overexpression showed that circMARK2 could be regulated by m^6^A modification in WT cells (Fig. 6G). Additionally, RIP assays revealed increased circMARK2 in HNRNPC precipitates post-METTL3 overexpression and decreased levels following ALKBH5 overexpression (Fig. S2G), underscoring the significance of m^6^A modification in the circMARK2-HNRNPC interaction.

Considering the largely unexplored area of circRNA subcellular trafficking and HNRNPC’s known role in facilitating the transport of m^6^A-modified mRNA between the nucleus and cytoplasm [42, 47], we investigated whether the export of m^6^A-modified circRNA is dependent on HNRNPC. Our nuclear and cytoplasmic fractionation experiments (Fig. 6H) and FISH (Fig. 6I) revealed that HNRNPC silencing significantly augmented nuclear retention of circRNA. However, overexpression of si-HNRNPC-insensitive Myc-tagged wild-type HNRNPC (Myc-WT-Ins), as opposed to the RRM truncated version (Myc-MUT-Ins) [48], effectively restored the impaired cytoplasmic export of circMARK2 resulting from HNRNPC depletion (Fig. 6H, I). These findings collectively suggest that HNRNPC binds to circMARK2 and facilitates its m^6^A-dependent export from the nucleus to the cytoplasm.

Subsequently, we explored the significance of m^6^A methylation on circMARK2 in the context of Wilms tumor (WT). Our results indicated that overexpression of circMARK2 led to an increase in both nuclear and cytoplasmic levels of circMARK2, especially in the cytoplasmic fraction (Fig. S2H). This overexpression was also associated with heightened m^6^A methylation levels (Fig. 6J) and enhanced proliferation and invasion of WT cells (Fig. 6K, L). Mutation of the GAACU m^6^A modification site within the circMARK2 overexpression construct, resulting in reduced m^6^A modification of circMARK2 (Fig. 6J), led to a decrease in WT cell invasion activity (Fig. 6K, L). These outcomes underscore the importance of m^6^A modification of circMARK2 in regulating the proliferation and invasion of WT cells.

### Nanomedicine consisting of C-SLN/si-circMARK2 complexes suppressed WT progression *in vivo*

Studies have suggested that the combination of the bioactive anticancer component and the gene would not only improve the transfection efficiency of the gene but also possess a synergistic effect of anticancer agents and gene therapies [49]. In line with these findings, our prior research demonstrated that nanomedicines comprising C-SLN/ASO-IGFL2-AS1 complexes and CS-EGCG/circSPIRE1 plasmid complexes specifically target renal cancer *in vivo* [50, 51]. We have reported that C-SLNs exhibit an average particle size of 247 ± 27 nm and a mean zeta potential of 1.4 ± 0.3 mV at near-neutral pH, optimal for cell endocytosis and binding to negatively charged ions, facilitating the controlled release of si-circMARK2 (siRNA). SiRNA binding assays indicated strong binding within C-SLN complexes at a mass ratio of 1:2.5 or higher, as evidenced by their near-invisibility (Fig. S3A). CCK8 assays on 293 T cells confirmed that C-SLN complexes exhibit minimal cytotoxicity at 120 μg/mL, a concentration double that required for high transfection efficiency (Fig. 7A). Further, we assessed the adsorption of lipo2000/FAM‐siRNA and C-SLN/FAM‐siRNA complexes in G401 and SK-NEP-1 cells using fluorescein (FAM)‐labeled siRNA (FAM‐siRNA) through confocal microscopy. Observations indicated superior internalization efficiency of C-SLN/FAM‐siRNA in WT cells compared to lipo2000/FAM‐siRNA after 6 h of incubation (Fig. 7B). At a total concentration of 60 μg/mL, C-SLN complexes achieved transfection efficiency comparable to liposomal-based lipo2000, with only modest changes observed at 120 μg/mL (Fig. 7C). Next, we validated the efficiency of circMARK2 knockdown by the C-SLN/siRNA. As confirmed by qPCR, the best C-SLN‐to‐siRNA mass ratio was 1:2.5 (Fig. 7D). To ascertain whether siRNA delivered by C-SLN could escape lysosomes and facilitate posttranscriptional gene silencing in the cytoplasm, we treated WT cells with C-SLN/siRNA for varying durations. Using LysoTracker staining and confocal microscopy, we observed the co-localization of red (LysoTracker) and green (C-SLN/FAM‐siRNA) fluorescence within cells after 1 h, indicative of FAM‐labeled siRNA in lysosomes. Over time, particularly at 6 h, the overlap between green and red fluorescence decreased, signifying the escape of C-SLN/siRNA from lysosomes (Fig. 7E).

**Fig. 7:** C-SLN/si-circMARK2 Nanocomplexes suppressed Wilms Tumor Progression *In Vivo*. **A** Cell cytotoxicity of C-SLN NPs complexing with siRNA was assessed by CCK8 assay and the percentage of viable cells was calculated relative to untreated control cells. Data represent mean ± S.D.; dot plots reflect data points from six independent experiments. **B** Confocal microscopy analysis of lipo2000/FAM‐siRNA or C-SLN/FAM‐siRNA distribution in WT cells. Green: fluorescein‐labeled siRNA; blue: Hoechst 33342‐stained nuclei. Scale bar, 10 µm. **C** Percentage of fluorescent cells analyzed by flow cytometry. Data represent mean ± S.D.; dot plots reflect data points from six independent experiments. **D** Optimal ratio of C-SLN to siRNA was determined through RT‐qPCR. **E** Representative confocal images of WT cells incubated using C-SLN/FAM‐siRNA under 37°C. Hoechst 33342 (blue) was used to stain nuclei, LysoTracker Red (red) was used to stain endo/lysosomes, while FAM (green) was used to label siRNAs. Scale bar, 10 µm. **F** Fluorescent fold change assay after treated by C-SLN composed nanomedicine. **G** Representative image of orthotopic patient-derived xenograft (PDX) tumor, HE and IHC assays. Scale bar, 100 µm. (*n* = 5 mice/group). **H** Serum levels of IFN-γ, IL-1β, TNF-α, IL-6, AST, ALT, CREA, and UREA after injections of PBS control, C-SLN, siRNA only or C-SLN/siRNA

Building on our previous demonstration of the stability and tumor-specific delivery of C-SLN composed nanomedicine in renal tumors *in vivo* [50], we further explored its therapeutic potential using an orthotopic patient-derived xenograft (PDX) model. The efficacy of C-SLN/siRNA in this model was monitored weekly through fluorescein *in viv*o imaging (Fig. 7F). Remarkably, the group treated with C-SLN/siRNA displayed superior therapeutic outcomes, evidenced by reduced tumor proliferation (Fig. 7G). Additionally, an increase in *LET-7* expression was noted in the C-SLN/siRNA group (Fig. 7G). To assess the potential side effects of C-SLN nanoparticles *in vivo*, we conducted a comprehensive blood serum analysis. The levels of inflammatory markers such as IL‐1β, IFN‐γ, IL‐6, and TNF‐α were found to be within normal ranges. Key hematological indicators, including urea, creatinine (CREA), alanine aminotransferase (ALT), and aspartate aminotransferase (AST) concentrations, also remained unaffected (Fig. 7H). Collectively, these findings suggest that C-SLN nanoparticles possess excellent biocompatibility, and their use in mediating circMARK2 silencing effectively suppresses the progression of Wilms tumor *in vivo*.

## Discussion

CircRNAs, known for their stability and prevalence, have garnered increasing attention in cancer research. Yet, their role in Wilms tumor (WT) remains less explored compared to other cancer types. This gap in understanding is particularly pressing given the modest 50% survival rate following WT relapse. There is a clear need for comprehensive research into the relationship between circRNA dysregulation and WT progression [7]. In our current study, we have discovered that circMARK2, a circRNA modified by N^6^-methyladenosine (m^6^A), plays a pivotal role in WT advancement. Our analysis reveals a consistent upregulation of circMARK2 in WT, which is strongly associated with disease progression and reduced patient survival. Employing patient-derived xenograft (PDX) models, our findings indicate that higher circMARK2 expression markedly accelerates WT progression. We have determined that the cytoplasmic export of circMARK2 is facilitated by HNRNPC, dependent on m^6^A modification. Crucially, this elevated cytoplasmic presence of circMARK2 significantly increases the stability of *LIN28B* mRNA via a circMARK2/IGF2BP2/*LIN28B* RNA–protein interaction complex, thereby enhancing the malignancy of WT cells. Clinically, elevated expressions of both circMARK2 and *LIN28B* are notably more common in advanced stages of WT, underscoring their potential as biomarkers for disease progression.

In this study, we selected both recurrent and primary WT samples for sequencing to capture a comprehensive spectrum of tumor biology. This approach enabled us to identify circRNAs like circMARK2, which are crucial for both tumor initiation and progression. Sequencing recurrent samples, known for their aggressive traits, alongside primary tumors allowed us to target circRNAs relevant to poor prognosis. We also intersected our data with the publicly available dataset GSE197046 to validate our findings across broader cohorts, enhancing the robustness and reproducibility of our results. This method ensured that identified circRNAs, particularly circMARK2, are consistently associated with disease progression and are viable therapeutic targets.

In recent years, circRNAs have emerged as significant players in cellular mechanisms, exhibiting diverse biological functions. Predominantly localized in the cytoplasm, circRNAs are often implicated as miRNA sponges, modulating gene expression, or as protein sponges through interactions with RNA-binding proteins (RBPs). While typically non-coding, certain circRNAs are known to undergo translation under specific conditions [5]. In the context of WT, the majority of circRNAs are understood to function as miRNA sponges [22]. A notable mechanism observed in colorectal carcinoma is the role of circNSUN2 in stabilizing *HMGA2* mRNA via an RNA–protein ternary complex formation [26], illustrating the potential of circRNAs to guide the targeted binding of RBPs to specific RNAs. In our study, mass spectrometry analysis identified IGF2BP2, a conventional RBP, as a major component in the circRNA-associated pull-down complex. This finding spurred our investigation into the guiding role of circRNAs in WT, marking the first exploration of this mechanism in this tumor type.

LIN28B, a critical RNA-binding protein, orchestrates gene expression by obstructing the maturation of *LET-7* family microRNAs (miRNAs), a process vital for cellular differentiation and growth regulation [52, 53]. This obstruction occurs as LIN28B binds to the terminal loop of primary and precursor LET-7 miRNAs, thereby inhibiting their maturation and allowing the expression of LET-7-targeted oncogenes, such as K-Ras and c-Myc [54, 55]. Notably expressed in pluripotent cells, LIN28B facilitates the maintenance of their proliferative and self-renewal capacities. Its expression is predominant in early embryogenesis, subsequently diminishing as cells undergo differentiation, inversely correlating with the maturation of *LET-7* miRNAs [56]. LIN28B proteins are highly expressed in early embryonic development but become down-regulated over time, while levels of mature *LET-7* family members rise as stem cells differentiate into specialized tissue types [55]. Overexpression of LIN28B is common in various tumor types and facilitates cellular transformation [57]. LIN28B has been linked to neuroblastoma [58], a pediatric tumor derived from neural crest tissues that fail to complete their differentiation program [59]. And Wilms tumor was reported to be caused by enforced overexpression of LIN28B as well [39]. Although increased LIN28B DNA copy number has been documented 25% of Wilms tumor [38], this alteration alone fails to account for the ubiquitous LIN28B overexpression observed across WT instances [39]. Our research posits a novel post-transcriptional regulation mechanism, wherein circMARK2, in conjunction with IGF2BP2, elevates LIN28B expression through forming circMARK2/IGF2BP2/*LIN28B* mRNA ternary complex, thereby elucidating an additional layer of complexity in the oncogenic landscape of WT.

N^6^-methyladenosine stands as the most prevalent internal modification on eukaryotic mRNA and various noncoding RNAs, including circRNAs [12]. This modification orchestrates a range of RNA metabolic processes, from splicing and localization to translation, stability, and degradation. Existing literature indicates that WT tissues express m^6^A regulators at higher levels than normal tissues, suggesting a link between altered RNA methylation patterns and WT pathogenesis [60]. Moreover, our earlier molecular epidemiological studies have uncovered associations between genetic variants in m^6^A-related enzymes like METTL14, ALKBH5 and FTO, and increased WT risk [18–21]. Despite these insights, the m^6^A modification of circRNAs in WT has not yet been explored. CircRNAs are typically considered byproducts of conventional linear mRNA splicing, arising within the nucleus. Nonetheless, their predominant localization in the cytoplasm implicates them in various biological roles [61]. Unraveling how circRNAs are transported from the nucleus to the cytoplasm is therefore crucial. Our work provides novel evidence that circMARK2's nuclear export in WT is m^6^A-dependent and facilitated by HNRNPC interaction. Coupled with the upregulated expression of m^6^A methylation enzymes in WT, circMARK2 is predisposed to cytoplasmic translocation, where it can engage in oncogenic activities that drive WT progression. The mechanism responsible for the increased overall expression of circMARK2 warrants further investigation.

## Conclusions

In summary, our research identifies circMARK2 as a key oncogenic circRNA and a potential prognostic marker for recurrent WT. It plays a vital role in the post-transcriptional enhancement of *LIN28B* mRNA stability, forming a complex with IGF2BP2 that augments the malignancy of WT cells. Crucially, circMARK2 emerges as a promising therapeutic target, opening new avenues for the treatment of WT, particularly for cases with a high risk of progression.

### Supplementary Information

Supplementary Material 1.

## Data Availability

All data associated with this study are presented in the paper or the Supplementary Data. Primers, probes, and RNAi target sequence were presented in Supplementary data 1. The materials that support the findings of this study are available from the corresponding author on reasonable request.
